# Integrating Optimized Multiscale Entropy Model with Machine Learning for the Localization of Epileptogenic Hemisphere in Temporal Lobe Epilepsy Using Resting-State fMRI

**DOI:** 10.1155/2021/1834123

**Published:** 2021-10-27

**Authors:** Xiaoxuan Fu, Youhua Wang, Abdelkader Nasreddine Belkacem, Qirui Zhang, Chong Xie, Yingxin Cao, Hao Cheng, Shenghua Chen

**Affiliations:** ^1^State Key Laboratory of Reliability and Intelligence of Electrical Equipment, Hebei University of Technology, Tianjin 300130, China; ^2^Key Laboratory of Electromagnetic Field and Electrical Apparatus Reliability of Hebei Province, Hebei University of Technology, Tianjin 300130, China; ^3^Department of Computer and Network Engineering, College of Information Technology, United Arab Emirates University, Al Ain 15551, UAE; ^4^Department of Medical Imaging, General Hospital of Eastern Theater of PLA, Nanjing 210002, China

## Abstract

The bottleneck associated with the validation of the parameters of the entropy model has limited the application of this model to modern functional imaging technologies such as the resting-state functional magnetic resonance imaging (rfMRI). In this study, an optimization algorithm that could choose the parameters of the multiscale entropy (MSE) model was developed, while the optimized effectiveness for localizing the epileptogenic hemisphere was validated through the classification rate with a supervised machine learning method. The rfMRI data of 20 mesial temporal lobe epilepsy patients with positive indicators (the indicators of epileptogenic hemisphere in clinic) in the hippocampal formation on either left or right hemisphere (equally divided into two groups) on the structural MRI were collected and preprocessed. Then, three parameters in the MSE model were statistically optimized by both receiver operating characteristic (ROC) curve and the area under the ROC curve value in the sensitivity analysis, and the intergroup significance of optimized entropy values was utilized to confirm the biomarked brain areas sensitive to the epileptogenic hemisphere. Finally, the optimized entropy values of these biomarked brain areas were regarded as the feature vectors input for a support vector machine to classify the epileptogenic hemisphere, and the classification effectiveness was cross-validated. Nine biomarked brain areas were confirmed by the optimized entropy values, including medial superior frontal gyrus and superior parietal gyrus (*p* < .01). The mean classification accuracy was greater than 90%. It can be concluded that combination of the optimized MSE model with the machine learning model can accurately confirm the epileptogenic hemisphere by rfMRI. With the powerful information interaction capabilities of 5G communication, the epilepsy side-fixing algorithm that requires computing power can be integrated into a cloud platform. The demand side only needs to upload patient data to the service platform to realize the preoperative assessment of epilepsy.

## 1. Introduction

Epilepsy is a chronic disease caused by abnormal neural discharges that could result in abnormal functions in the central nervous system. This disease could adversely impact the patient's quality of life and may even lead to death. The positive hippocampus on the structural magnetic resonance imaging (sMRI) is the most common pathological marker in the medial temporal lobe epilepsy (mTLE). It is also an indicator of epileptogenic hemisphere. The paroxysmal discharges might propagate to the large-scale brain networks and lead to metabolic dysfunction or structural changes in the distal brain regions connected with the primary lesion. Surgical treatment is a preferred method for intractable epilepsy, and more than 70% of focal epilepsy patients had experienced favorable postsurgical seizure control and exhibited the most positive therapeutic effect [1,2]. The precise assessments such as epileptogenic hemisphere, epileptogenic zone, and propagation pathway are important prior to the surgery [3]. They can not only help remove abnormal brain tissue, but also avoid damage to other functional areas such as language and memory as much as possible. In particular, the confirmation of the epileptogenic hemisphere is a basis. Integrating machine learning to locate epilepsy hemispheres has become a current research hotspot. Jin et al. [4] used magnetoencephalograms (MEG) to find the biomarker of functional connectivity (FC) to predict the epileptic hemisphere by support vector machine (SVM) with a classification rate of 76.2%. Barron et al. [5] had developed an automatic computer-aided diagnosis tool, which can determine the epileptogenic hemisphere by Positron Emission Computed Tomography (PET), with an accuracy rate of 82%.

Resting-state functional magnetic resonance imaging (rfMRI), a modern technology, has gained prominence for the task of revealing the pathological functions in the different regions in the brain, with some advantages such as noninvasive, objective, quick (in less than 15 min), conformable, and highly adaptive. It is therefore of great clinical value for pre- and postoperative monitoring and treatment of neurological diseases [6–8]. Now, based on rfMRI data, Zheng et al. could locate the the epileptogenic hemisphere with an accuracy of 83.8% by the combination of FC and SVM [9]. Therefore, the classification rate needs to be improved. As the neurological diseases affect brain functions on multiple temporal and spatial scales, Costa et al. [10] proposed the multiscale entropy (MSE) model that combined the sample entropy with the time scale to jointly uncover the complex characteristics under different physiological states. It is now extensively adopted for investigating neural signals [11–17], such as electroencephalography (EEG) [18–21], MRI [22,23], and magnetoencephalography (MEG) [24]. With regard to complexity, the MSE algorithm can reveal the physiological, pathological, and functional changes in the brain. The nonlinearity of the rfMRI signal of an epileptic patient is higher than corresponding signal for a healthy individual [25, 26], and thus the entropy model has the potential to evaluate the functions in an epileptic brain.

However, the selection of parameter dimension *m* and similarity *r* of MSE model depends on experiences and lacks an objective basis from the past to the present. The values of these parameters in different studies in the pertinent literature were *m* = 1, *r* = 0.35 [27], *m* = 1, *r* = 0.3 [28], *m* = 1, *r* = 0.35 [29], and *m* = 2, *r* = 0.6 [30]. Evidently, there is a problem of no uniform parameter standard or specification for MSE to process biomedical signals, leading to subjectivity in the entropy calculation. In this study, for the task of localizing the epileptogenic hemisphere, we developed an optimization algorithm for the parameters of the MSE model based on the rfMRI data scanned on the mTLE patients with a positive indicator in the hippocampal formation on sMRI. The hemisphere of these patients was considered epileptogenic in a clinic. The proposed approach for selecting the parameters of the entropy model in the epileptic rfMRI is demonstrated to be objected.

We investigated the extant literature on parameter optimization, with the help of the sensitivity analysis indexes-receiver operating characteristic (ROC) curves and the area under the ROC curve (AUC). After the parameters of epileptic entropy model were optimized, the entropy model was employed to extract the sensitive functional image markers, whose entropy values were considered as feature vectors and input to the support vector machine (SVM) to assess the feasibility and accuracy of optimal entropy model. Since the SVM is a supervised machine learning model and needs to be run on correctly labeled samples, the rfMRI data of mTLE patients with the positive hippocampus of sMRI were analyzed using the SVM. The study flowchart is shown in Figure 1.

## 2. Materials and Methods

### 2.1. Data Acquisition

The rfMRI data of 20 mTLE were collected from the Department of Medical Imaging, General Hospital of Eastern Theater of PLA, China, including nine males and 11 females, aged 19−33 (25.7 ± 3.7) years, who underwent a routine preoperative evaluation to localize the epileptogenic discharge areas. There were 10 patients (left group) with the positive indicator on the left hippocampus and the other 10 patients (right group) on the right hippocampus on sMRI.

When scanning, participants were asked to keep their eyes closed, stay awake, and think nothing. All rfMRI data were collected using a 3.0 T Magnetom Vision plus MR-scanner (Siemens, Erlangen Germany) and blood-oxygen-level-dependent (BOLD)-sensitive echo plane imaging sequence. The parameters were set as follows: TE/TR = 30/2000 ms, FA = 90°, FOV = 240 mm, voxel size = 3 × 3 × 3 mm3, and slice thickness = 4 mm [31]. This study was approved by the Medical Ethics Committee of General Hospital of Eastern Theater of PLA in China, and the patients were provided with the requisite information and signed the informed consent form.

### 2.2. Data Processing

Data processing was accomplished using both pre- and postprocessing techniques.

All rfMRI data were preprocessed using FMRIB software [32,33]. Preprocessing procedure and quality inspection (framewise displacement (FD) < 0.2 mm) were conducted at Martinos Center for Medical Imaging, Harvard Medical School, USA [34,35]. The processing station used was Intel Xeon Sliver 4112 × 16 with the operating system of Centos 7.6, and the preprocessing time was about 15 hours for each subject.

The different steps for data preprocessing can be enumerated as follows: (1) removal of the first four acquisition time series to stabilize the signal, (2) slice timing correction (SPM2, Wellcome Department of Cognitive Neurology, London, UK), (3) rigid body correction for head motion with the FMRIB software library package (http://fsl.fmrib.ox.ac.uk/fsl) [36], (4) normalization for global mean signal intensity across runs and registration of the signal to the standard space of Montreal neurological institute, and (5) band-pass temporal filtering (0.01Hz−0.08 Hz).

During postprocessing, data were projected to the brain region AAL1 (Anatomical Automatic Labeling, Version 1) using DPABI of MATLAB R2018b in the Windows V.10 operating system. The whole brain of each subject was divided into 116 brain regions, and each brain region has 246 time points in a 490 s time length. The overall postprocessing time was about 14 hours. Among 116 brain regions, 90 cortical cortex regions were examined in this study.

### 2.3. MSE Model

For one-dimensional N-length discrete time series {*x*_1_,  *x*_2_,  *x*_3_,…,  *x*_*N*_}, the length of each coarse-grained time series {*y*_*j*_^*τ*^} is equal to the length of original time series divided by the time scale *τ* in the following formula:

(1) $$\begin{array}{c} y_{j}^{\tau }\;=\;\frac{1}{\tau }\sum_{i\;=\;\left(j\;–\;i\right)\tau \;+\;1}^{j\tau }x_{i}, \end{array}$$

where 1 ≤ *j* ≤ *N*/*τ*, *τ* is the scale factor, and the length of {*y*_*j*_^*τ*^} is *L* = *N*/*τ*.

Then, a set of m-dimension vectors (m is embedding dimension) Ym(i) are formed: Ym(i) = {yi + *k*, 0 ≤ *k* ≤ *m* − 1}. For each *i* value, its distance from other value *j* is calculated, that is, the distance between Ym(i) and Ym(*j*) is shown in the following formula:

(2) $$\begin{array}{c} d\left[Ym\left(i\right),Ym\left(j\right)\right]=\max\left|\;y\left(i+k\right)-y\left(j+k\right)\right|\left(0\leq k\leq m-1,i,j=1-L-m+1,I\neq j\right). \end{array}$$

Setting the tolerance threshold (i.e., similarity factor) *r* (*r* ＞ 0), the number Bm(i) of d[Ym(i), Ym(*j*)] < *r* is calculated for each *i* value, and the ratio to the total distance can be obtainable by *C*_*τ*_^*m*^(*r*) =*B*^*m*^(*i*)/*L* – *m*. And then, the average of *C*_*τ*_^*m*^(*r*) is shown as follows:

(3) $$\begin{array}{c} C^{m}\left(r\right)=\;\frac{1}{L\;–\;m\;+\;1}C_{\tau }^{m}\left(r\right). \end{array}$$

Likewise, for *m* + 1 dimension, the average can be derived as

(4) $$\begin{array}{c} C^{m\;+\;1}\left(r\right)\;=\;\frac{1}{L\;–\;m}\sum_{i=1}^{L\;-\;m}C_{\tau }^{m\;+\;1}\left(r\right). \end{array}$$

Given that the sequence length *L* is a finite value, the entropy with *L* can be estimated, denoted as MSE using the followig formula:

(5) $$\begin{array}{c} \text{MSE}\left(\tau ,m,r\right)=–\;\ln\left[\frac{C^{m\;+\;1}\left(r\right)}{C^{m}\left(r\right)}\right]. \end{array}$$

The size of entropy value is related to the repeatability of time series. The larger the entropy value, the greater the complexity, and vice versa.

As the three parameters interacted with each other, they needed to participate in the optimization of each parameter. The dimension *m* was optimized at first, followed by the optimization of similarity *r* and time scale *τ*.

In general, the accuracy of entropy evaluation improves with the increase in the number of vector matches in dimension *m* and *m* + 1. Using BOLD signal, the entropy can be accurately estimated in the time length of 10 m−20 m [37]. On the basis of the time point length of data (246 time points), the dimension *m* could be estimated in a range of 1−2; that is, the optimization of dimension *m* would be conducted by *m* = 1 or 2.

According to previous analysis, the range of similarity *r* could be selected from 0.05 to 0.6 [27–30,38,39]. However, there were some invalid values in the entropy calculation at *r* = 0.05–0.3. Accounting for a short length of time series in this study, the similarity *r* could not be too small. Thus, the similarity *r* could be within the range of 0.3–0.6. We conducted the entropy calculation with a step size of 0.02. As usual, the time scale *τ* could be optimized in a range of 1−5 with a step size of 1.

Here, both ROC curve and AUC value were used to assess the optimization effect. Both these values converged during the evaluation. That is, the more the ROC curve was above the reference line; the greater the AUC value was, and the better the classification effect was. However, ROC curves below the reference signified the classification insignificance. When the ROC curve of a brain area was above the reference line, this brain area could be considered sensitive to the epileptogenic hemisphere. Conversely, when the ROC curve of a brain area was around the reference line, this brain area could be considered insensitive to the epileptogenic hemisphere. The optimal procedures were individually conducted for all the 90 brain areas. For the sake of explanation, the specific brain regions were taken as examples, such as left superior frontal gyrus, medial (SFGmed.L), right superior parietal gyrus (SPG.R), left cuneus (CUN.L), and left thalamus (THA.L).

The brain area with a significant difference (*p* < .05) of the optimized entropy values between the two groups was considered to be the functional biomarked sensitive to epileptogenic hemisphere. The statistics were performed by *t*-test through software of Statistical Package for the Social Science (SPSS) (IBM SPSS Statistics 21; USA). The ROC curve and the AUC value were used to verify the biomarkers. BrainNet Viewer was employed to visualize the biomarkers (http://www.nitrc.org/projects/bnv/) [40].

### 2.4. SVM

SVM-based machine learning model is not easily influenced by the dimension of data and the limitation of the sample size. In particular, it could simultaneously minimize the empirical classification error and maximize the geometric margin. It is thus better than other conventional machine learning models.

The optimized entropy values of functional biomarked areas were considered to be the feature vectors input into the SVM model. The mTLE patients in the left group were marked as ‘‘1,” and those in the right group were marked as “0”.

The optimized MSE values of 20 subjects were taken as the input to the SVM model. The data from 8 subjects were used as the training set and from 12 subjects as the testing set. In the SVM model, the radial basis function (RBF) was considered as the kernel function, and the kernel parameter *σ* was replaced with the proportional parameter *g* =1/2*σ*^2^ to form a set of parameter pairs (*C*, *g*). Ranges of both these parameters were set as [−10,10] with a step size of 0.2. The optimal values of *C* and *g* were confirmed by the grid search method and then used to build the training model and the test sets.

The leave-one-out cross-validation (LOOCV) is often used to test the accuracy of the algorithm model, and its sample utilization is very high; thus, it is highly suitable for small samples analysis. If there are N sample data, then N − 1 samples constitute the training data, and the remainder constitutes the testing data. Therefore, the mean accuracy of N times (*N* = 20) can be used to evaluate the classification accuracy.

## 3. Results and Discussion

### 3.1. Parametric Optimization of MSE Model

After preprocessing, the length of BOLD signal was 246 time points in the mTLE. Thus, the value of *m* can be 1 or 2. According to the previous studies, the optimized parametric spaces were confirmed in a range of *r* = 0.3–0.6 (step size of 0.02) and *τ*  = 1−5 (step size of 1).

#### 3.1.1. Optimization of Dimension m and Similarity *r*

In Figure 2, the dimension *m* was optimized by the number of significant brain regions between two groups (*p* < .05) when the time scale *τ*  = 1−5 with a step size of 1 and the similarity *r* = 0.3–0.6 with a step size of 0.02. It was found that the number of significant brain regions of *m* = 1 was generally greater than that of *m* = 2. Therefore, *m* = 1 was selected as the optimization parameter. Moreover, the difference is significant at *τ*  = 2 and *τ*  = 3, so the optimization parameter of *τ* might be derived from *τ*  = 2−3.

Additionally, it was found that the number of significant brain regions at *r* = 0.54–0.6 were generally greater than other *r* values. That is, the optimization value of similarity *r* could be derived from 0.54–0.6.

By setting *m* = 1 and *r* = 0.54–0.6 (step size of 0.02) fixed, the ROC curves of left superior frontal gyrus, SFGmed.L, SPG.R, CUN.L, and THA.L at different *r* values were taken as examples in Figure 3. The results of *τ*  = 2 and *τ*  = 3 are similar; therefore, only the result of *τ*  = 3 is shown here; it was found that the ROC curves of SFGmed.L and SPG.R were all above the reference lines, indicating that SFGmed.L and SPG.R could be considered sensitive to the epileptogenic hemisphere. Conversely, the ROC curves of CUN.L and THA.L were around the reference line and thus insensitive to the epileptogenic hemisphere.

The AUC value of each brain region and the corresponding similarity factor (*r*) are presented in Table 1. Evidently, the AUC values of SFGmed.L and SPG.R were the largest when *r* = 0.56 (yellow line in Figures 3(a) and 3(b)), which indicates that *r* = 0.56 was the optimized value.

#### 3.1.2. Optimization of Time Scale *τ*

Setting *m* = 1, *r* = 0.56, and *τ*  = 1−5, the obtained ROC curves of left insula (INS.L), left Rolandic operculum (ROL.L), CUN.L, and left superior frontal gyrus, dorsolateral (SFGdor.L) at different *τ* values are shown in Figure 4.

The AUC value of each brain region by time scale *τ* is presented in Table 2, and it was found that the AUC values of INS.L and ROL.L were the largest at *τ*  = 3 (green line in Figure 4), suggesting that *τ*  = 3 was the optimized value.

In summary, the optimized parameters of MSE model derived from the epileptic rfMRI data were *m* = 1, *r* = 0.56, and *τ*  = 3.

### 3.2. Feature Vector

With the optimized parameters *m* = 1, *r* = 0.56, and *τ*  = 3, a total of nine brain regions sensitive to the epileptogenic hemisphere were obtained by the intergroup entropy values (*p* < .01), that is, left Rolandic operculum (ROL.L, AAL17), right Rolandic operculum (ROL.R, AAL18), left superior frontal gyrus, medial (SFGmed.L, AAL23), left insula (INS.L, AAL29), right insula (INS.R, AAL30), left superior parietal gyrus (SPG.L, AAL60), left precuneus (PCUN.L, AAL67), left caudate nucleus (CAU.L, AAL73), and right temporal pole: superior temporal gyrus (TPOsup.R, AAL84). The projection of nine brain regions on the cortical surface and their ROC curves are depicted in Figure 5.

### 3.3. Leave-One-Out Cross-Validation

The MSE values of nine biomarked brain regions were used as feature vectors input for SVM-based classification. All classification rates (CR) of 20 times are shown in Table 3. The validity of MSE model is verified using leave-one-out cross-validation (LOOCV), and the mean classification accuracy of LOOCV was found to be 95%.

### 3.4. Discussion

#### 3.4.1. MSE Model to Image the Brain

From a theoretical perspective, the MSE model can comprehensively analyze the dynamical changes of signals by calculating the complexity of time series [19]. In addition, because epilepsy is a dynamical disease, the MSE model has the potential to be utilized in the assessment of dysfunction in epilepsy [41]. Finally, since the functional connectivity of Pearson correlation (FC) is a conventional index, its relationship between FC and entropy would provide support for the optimized MSE to image the functional brain. Wang et al. [42] affirmed that the relationship between MSE value of the rfMRI time series and FC depended on the length of time series and the size of time scale *τ*. By the MSE model of the rfMRI data, Yang et al. [27] found that the people with different cognitive scores can be fairly distinguished using a MSE-based model. William et al. [43] examined if the MSE model of EEG data can distinguish the absence epilepsy patients from healthy control with high accuracy (>95%).

#### 3.4.2. Functional Biomarker of TLE

At present, the mTLE lesions are identified by certain biomarked brain regions including the insula, bilateral cingulate gyrus, and precuneus [4,9,44]. By considering the healthy people as a control, Zhou et al. [45] found that the left middle temporal gyrus, right middle frontal gyrus, and the left anterior central gyrus were significantly different in temporal lobe epilepsy by the entropy values of the rfMRI data. In addition, by the anatomical connectivity between the left and right hemispheres in the temporal lobe epilepsy, a different connectivity pattern was observed in the cortical-limbic network and cerebellum [46]. These biomarked brain regions have a great intersection with the current study.

#### 3.4.3. Analysis in Healthcare 5.0

With the powerful information interaction capabilities of 5G communication, the epilepsy positioning algorithm combined with multiscale entropy can be integrated into a software package in the future to build a cloud platform server for epilepsy positioning. Since the lateralization software combined with the multiscale sample entropy model requires a lot of computing power, the computing power can be provided by the server, and the user only needs to upload the patient's fMRI image to the cloud platform server to obtain the lateralization result.

## 4. Conclusion

Through the optimized MSE model, a total of nine landmarks sensitive to the epileptogenic hemisphere of temporal lobe epilepsy could be estimated in the left Rolandic operculum, right Rolandic operculum, left superior frontal gyrus, medial, left insula, and so on. The mean CRs attained through LOOCV were 95%, respectively. This work underlines the importance of an optimized entropy model and presents an automated detection algorithm for rfMRI to aid the preoperative assessment of epilepsy.

## Figures and Tables

**Figure 1:** Study flowchart.

**Figure 2:** Optimal value of parameter (*m*) estimated by number of brain regions with intergroup significant difference (*p* < .05). (a)*τ*  = 1; (b)*τ*  = 2; (c)*τ*  = 3; (d)*τ*  = 4; (e)*τ*  = 5; (f) average number of brain regions over time scale *τ*.

**Figure 3:** Effects of similarity (*r*) on the epileptogenic hemisphere classification of a single brain area displayed by ROC curves, setting *m* = 1 and *τ*  = 3 constant, similarity (*r*) varying from 0.54 to 0.6 with a step of 0.02. (a) SFGmed.L; (b) SPG.R; (c) CUN.L; (d) THA.L.

**Figure 4:** Effects of scale factor *τ* on the epileptogenic hemisphere classification of a single brain area displayed by ROC curves, setting *m* = 1, *r* = 0.56 constant and time scale (*τ*) variable from 1 to 5 with a step of 1. (a) INS.L; (b) ROL.L; (c) CUN.L; (d) SFGdor.R.

**Figure 5:** Biomarker brain regions indicated by a brain template in the software of BrainNet Viewer (a) and its ROC curves at optimized parameters (*m* = 1, *r* = 0.56, and *τ*  = 3) (b).

**Table 1:** AUC value of each brain region by similarity (*r*).

Similarity r	SFGmed.L	SPG.R	CUN.L	THA.L
*r* = 0.54	0.92	0.89	0.53	0.65
*r* = 0.56	0.93	0.90	0.53	0.69
*r* = 0.58	0.89	0.86	0.50	0.56
*r* = 0.60	0.89	0.90	0.54	0.61

**Table 2:** AUC value of each brain region by time scale *τ*.

Time scale *τ*	INS.L	ROL.L	CUN.L	SFGdor.R
*τ*=1	0.43	0.46	0.43	0.38
*τ*=2	0.8	0.84	0.63	0.55
*τ*=3	0.83	0.91	0.53	0.54
*τ*=4	0.45	0.67	0.47	0.40
*τ*=5	0.62	0.65	0.41	0.59

**Table 3:** Classification by LOOCV.

ID	1	2	3	4	5	6	7	8	9	10
Result	T	T	T	T	T	T	T	T	T	T
ID	11	12	13	14	15	16	17	18	19	20
Result	F	T	T	T	T	T	T	T	T	T

T: prediction is converge to diagnose; F: prediction is reversal to diagnose.

## Data Availability

Due to the privacy protection of patient data, the availability of original data cannot be provided.
